The article "Secondary bile acids mediate high-fat diet–induced upregulation of R-spondin 3 and intestinal epithelial proliferation" was retracted in 2024. Reasons: fabricated or falsified data; an official misconduct investigation.

# Secondary bile acids mediate high-fat diet–induced upregulation of R-spondin 3 and intestinal epithelial proliferation

**DOI:** 10.1172/jci.insight.148309

**Published:** 2022-10-10

**Authors:** Ji-Yao Li, Merritt Gillilland, Allen A. Lee, Xiaoyin Wu, Shi-Yi Zhou, Chung Owyang

**Affiliations:** Division of Gastroenterology and Hepatology, Department of Internal Medicine, University of Michigan, Ann Arbor, Michigan, USA.

**Keywords:** Gastroenterology, Colorectal cancer, Mouse stem cells

## Abstract

A high-fat diet (HFD) contributes to the increased incidence of colorectal cancer, but the mechanisms are unclear. We found that R-spondin 3 (Rspo3), a ligand for leucine-rich, repeat-containing GPCR 4 and 5 (LGR4 and LGR5), was the main subtype of R-spondins and was produced by myofibroblasts beneath the crypts in the intestine. HFD upregulated colonic Rspo3, LGR4, LGR5, and β-catenin gene expression in specific pathogen–free rodents, but not in germ-free mice, and the upregulations were prevented by the bile acid (BA) binder cholestyramine or antibiotic treatment, indicating mediation by both BA and gut microbiota. Cholestyramine or antibiotic treatments prevented HFD-induced enrichment of members of the Lachnospiraceae and Rumincoccaceae, which can transform primary BA into secondary BA. Oral administration of deoxycholic acid (DCA), or inoculation of a combination of the BA deconjugator *Lactobacillus plantarum* and 7α-dehydroxylase–containing *Clostridium scindens* with an HFD to germ-free mice increased serum DCA and colonic Rspo3 mRNA levels, indicating that formation of secondary BA by gut microbiota is responsible for HFD-induced upregulation of Rspo3. In primary myofibroblasts, DCA increased Rspo3 mRNA via TGR5. Finally, we showed that cholestyramine or conditional deletion of Rspo3 prevented HFD- or DCA-induced intestinal proliferation. We conclude that secondary BA is responsible for HFD-induced upregulation of Rspo3, which, in turn, mediates HFD-induced intestinal epithelial proliferation.

## Introduction

Epidemiologic studies have linked obesity with increased risk for colorectal adenomas and cancer (1–3). Although the incidence is highest in industrialized countries, incidence is increasing in developing countries as they adopt a Western lifestyle (4). Environmental factors, particularly a high-fat diet (HFD), are believed to mediate this increased risk for colorectal cancer (5). However, the mechanism(s) by which intestinal stem cells sense dietary signals in the intestinal microenvironment that result in intestinal epithelial cell proliferation are still unclear.

The leucine-rich, repeat-containing GPCRs (LGRs) are critical for survival of intestinal stem cells and have been strongly implicated in the pathogenesis of colorectal cancer (6, 7). LGR5 is a stem cell marker in the small intestine and colon, whereas LGR4, a closely related homolog, is required for maintenance of intestinal stem cells (8, 9). Accumulating evidence suggests that an HFD may stimulate LGR5^+^ intestinal stem cell proliferation, which has been shown to be the colorectal cancer cells of origin in mouse models (10, 11). In addition, LGR4 and LGR5 are overexpressed in colorectal cancer and are associated with poorer outcomes (12–14). Meanwhile, nonsense mutations in LGR4 were associated with lowered body weight, and functional missense mutations in LGR4 were linked with increased obesity and metabolic complications (15, 16). This suggests that LGR plays a pivotal role in regulating both obesity and colorectal cancer risk.

The article "Secondary bile acids mediate high-fat diet–induced upregulation of R-spondin 3 and intestinal epithelial proliferation" was retracted in 2024. Reasons: fabricated or falsified data; an official misconduct investigation.

R-spondins (Rspos) are a family of 4 secreted proteins (Rspo1 through Rspo4) that potentiate the Wnt signaling pathway, which is critical for normal development and survival of intestinal stem cells. All 4 Rspo proteins function as ligands for LGR4 and LGR5, with resultant activation of the Wnt pathway (17–19). The Wnt signaling pathway regulates the proliferative activity of intestinal crypt cells, and mutations that activate the Wnt pathway are seen in up to 90% of colorectal cancers (20–22). Rspo proteins markedly potentiate Wnt signaling pathways and drive stem cell expansion (23, 24). One study demonstrated gain-of-expression gene fusion involving Rspo2 and Rspo3 in 10% of human colorectal cancers (25). Notably, Rspo gene fusions were mutually exclusive of adenomatous polyposis coli (APC) mutations, which suggests that Rspo activation can substitute as an alternative driver for colorectal cancer. There is little information on how dietary and environmental factors regulate Rspo expression and function. Our preliminary studies show that Rspo3 is upregulated in the gut mucosa after a high-fat feeding in rats. However, the source of Rspo3 in the intestine and its role in regulating intestinal stem cell fate related to nutrient cues is not clear. In this study, we aimed to determine the source of Rspo3 in the intestine and to investigate its role in HFD-induced intestinal proliferation and the mechanisms responsible for upregulation of Rspo3 in response to an HFD.

## Results

### Rspo3 is present mainly in the intestinal myofibroblasts.

Using reverse transcription PCR (RT-PCR), we showed that both Rspo1 and Rspo3 were expressed in mouse and rat intestines (Figure 1, A and B). However, Rspo3 expression was more than 5-fold higher than Rspo1 in both small intestine and colon. Rspo2 and 4 were not detectable, indicating that Rspo3 is the major Rspo subtype in the intestines. Similarly, Rspo3 was the sole subtype detected in human colon biopsy specimens, whereas Rspo1-4 were not detected in human colonoids, indicating they are not produced by the epithelium (Figure 1C). Because Rspo3 is the major subtype of Rspo in the intestines, we focused on Rspo3 for further investigation. ISH revealed that, in rat intestine, Rspo3 mRNA was present exclusively in the lamina propria, beneath the crypt (Figure 1D). Double ISH showed that in rat small and large intestines, approximately 70% of Rspo3 colocalized with cells expressing the myofibroblast marker α–smooth muscle actin (α-SMA) beneath the crypt, indicating that myofibroblasts close to the crypt are the main source of Rspo3. Approximately 20% of Rspo3 colocalized with cells expressing the fibroblast marker vimentin, whereas approximately 10% of Rspo3 was expressed by unknown cell types in the lamina propria (Figure 1, E–G). Similar observations were found in the mouse colon (Figure 1H).

The article "Secondary bile acids mediate high-fat diet–induced upregulation of R-spondin 3 and intestinal epithelial proliferation" was retracted in 2024. Reasons: fabricated or falsified data; an official misconduct investigation.

### Rspo3 is upregulated by HFD feeding.

Mice fed an HFD (58 kcal% fat) had increased mRNA expression of colon Rspo3, LGR4, and LGR5 by 130%, 60%, and 62%, respectively (Figure 2A), whereas Rspo1 levels did not change. Moreover, levels of β-catenin, the key molecule in the signal transduction pathways for LGR4 and LGR5, were increased by 65%. Consistently, immunofluorescence showed that the protein levels of Rspo3, LGR4, LGR5, and β-catenin were increased in the mouse colon after HFD feeding (Supplemental Figure 1, A–D; supplemental material available online with this article; https://doi.org/10.1172/jci.insight.148309DS1).

Similarly, the expression of these genes was upregulated in the rat colon as the result of an HFD (Figure 2C), and Rspo3 mRNA expression was also increased in rat ileum as the result of HFD feeding (Supplemental Figure 2A). Although we detected by RT-PCR the expressions of low levels of Wnt3 and Wnt6 and high levels of Wnt receptors Frizzled 4 (Fzd4), Fzd6, and Fzd7 in mouse colon, none of them was changed by an HFD as determined by quantitative PCR (qPCR) (data not shown). These data indicate an HFD enhances the Wnt pathway via the Rspo3-LGR system.

Given the low fiber content in high-fat chow, we next investigated whether the low fiber content in an HFD contributes to gene upregulation of Rspo3. Addition of fermentable or nonfermentable fiber to HFD showed no significant effect on HFD-induced gene upregulation of Rspo3 (Supplemental Figure 2B). This indicates that the high fat content, rather than low fiber, in HFD is responsible for the Rspo3 gene upregulation.

We next investigated whether other food components have any effect on Rspo3 gene expression. Although a high-protein diet (60% kcal protein) and a diet high in red meat (40% beef) induced Rspo3 mRNA levels in mouse colon by 31% and 63%, respectively, they were both less potent at inducing Rspo3 expression compared with an HFD (Figure 2B). Meanwhile, a high-carbohydrate diet had no effect on Rspo3 levels. These data indicate that dietary fat is the strongest inducer of Rspo3 gene expression.

The article "Secondary bile acids mediate high-fat diet–induced upregulation of R-spondin 3 and intestinal epithelial proliferation" was retracted in 2024. Reasons: fabricated or falsified data; an official misconduct investigation.

We previously demonstrated that an HFD increased the level of circulating bile acids (BAs) (26). We thus examined whether elevated levels of BAs might be responsible for the upregulation of Rspo3, LGR4, and LGR5 gene expression. Concurrent administration of a BA binder, cholestyramine, prevented HFD-induced upregulation of Rspo3, LGR4, LGR5, and β-catenin gene expression in rat colon (Figure 2C). Cholestyramine treatment also prevented the upregulation of Rspo3 in rat ileum (Supplemental Figure 2A). These data indicate that BAs are responsible for HFD-induced upregulation of Rspo3, LGR4, LGR5, and β-catenin gene expression.

Given the importance of the effect of diet on the indigenous microbiota (27) as well as the microbiota’s role in regulating the BA pool (28), we next investigated whether the gut microbiota were involved in regulating gene expression of Rspo3, LGR4, LGR5, and β-catenin. In germ-free mice, eating an HFD for 2 weeks did not induce the upregulation of Rspo3, LGR5, LGR5, or β-catenin genes (Figure 2D). However, oral gavage of germ-free mice with mouse fecal microbiota resulted in upregulation of colon Rspo3 by 80% compared with germ-free mice after 2 weeks of eating an HFD (Figure 2E). Similarly, in rats, oral administration of antibiotics (namely, ampicillin, vancomycin, neomycin, and metronidazole) (29) as well as an HFD for 2 weeks attenuated the HFD-induced upregulation of Rspo3 gene expression (Figure 2F). These data suggest that the gut microbiota are also involved in upregulation of the Rspo3–LGR system in the colon.

### BA binders or antibiotic treatment normalizes dysbiosis caused by an HFD.

To explore whether BAs mediate the relationship between the gut microbiota and the Rspo3–LGR system in the gut, we performed 16S rRNA gene sequencing on rat fecal samples, using the MiSeq Illumina sequencing platform. HFD resulted in an enrichment of 38 operational taxonomic units (OTUs). Notably, 26 of the 38 OTUs (67%) were members of the Lachnospiraceae and Rumincoccaceae, which are 2 families of bacteria encoding major BA enzymes required for transforming primary BAs into secondary BAs (30). These microbial changes induced by an HFD were prevented by cholestyramine treatment in rats (Figure 3, A and B). Similarly, antibiotic treatment significantly reduced the abundance of 77 OTUs enriched by an HFD (Figure 4, A and B, and Supplemental Figure 3, A and B) with 45 of these 77 OTUs (58.4%) constituting members of the Lachnospiraceae and Ruminococcaceae. Antibiotic treatment also decreased OTU richness and community diversity (Supplemental Figure 3, C and D).

The article "Secondary bile acids mediate high-fat diet–induced upregulation of R-spondin 3 and intestinal epithelial proliferation" was retracted in 2024. Reasons: fabricated or falsified data; an official misconduct investigation.

It has been reported that levels of deoxycholic acid (DCA), a major, free secondary BA, are increased, whereas those of cholic acid (CA) and ursodeoxycholic acid (UDCA) are decreased, lithocholic acid (LCA) levels tend to decrease, and chenodeoxycholic acid (CDCA) levels in mouse serum do not change after HFD (31). Consistent with this report, our BA profiling results showed HFD resulted in significantly elevated mouse serum DCA levels, but LCA levels were lower than the detectable limit; CA and UDCA levels decreased but with no statistical significance (Supplemental Figure 4A), suggesting HFD promotes the transformation of CA into DCA. Thus, we focused on the effect of DCA on Rspo3 gene expression. In germ-free mice, oral administration of DCA with HFD increased Rspo3 mRNA in the colon (Supplemental Figure 2C).

BAs are conjugated to either taurine or glycine (bile salts) when secreted from the liver to the small intestine (32). In the intestine, gut bacteria that contain the enzymes known as bile salts hydrolases (BSHs) remove taurine and glycine from bile salts to form free primary BAs (i.e., CA and CDCA). The process is called deconjugation. In the colon, free primary BAs are further transformed into secondary BAs (i.e., DCA and LCA) by bacteria that contain 7α-dehydroxylase. A prerequisite for these transformations is deconjugation (33, 34). To further investigate the role of bacterial transformation of BAs by gut bacteria in HFD-induced upregulation of Rspo3 gene expression, we inoculated germ-free mice with either *Lactobacillus plantarum* (10^8^ CFU), which contains BSH for bile salt deconjugation (35), or *Clostridium scindens* (10^8^ CFU), which contains 7α-dehydroxylates for BA transformation (36), or a combination of both *L*. *plantarum* and *C*. *scindens* (double inoculations), and fed the mice an HFD for 2 weeks. The successful colonization of *L*. *plantarum*, *C*. *scindens*, or both in germ-free mouse gut was validated at the end of 2 weeks by qPCR using bacterial species–specific primers and mouse fecal DNA. With double inoculations, *C*. *scindens* showed a reduced efficiency of colonization in some mice compared with single inoculation, but both *L*. *plantarum* and *C*. *scindens* were detected (Supplemental Figure 5, A and B). We showed that an HFD did not induce upregulation of Rspo3 in the colon of mice inoculated with either *L*. *plantarum* or *C*. *scindens* alone; however, in double-inoculated mice, HFD induced upregulation of Rspo3 significantly (Supplemental Figure 2C). Serum DCA was not detectable in mice inoculated with either *L*. *plantarum* or *C*. *scindens* alone, but serum DCA levels were elevated in double-inoculated mice (Supplemental Figure 4A), suggesting that the transformation of primary to secondary BAs is critical for HFD-induced upregulation of Rspo3. We also observed an elevated level of α-muricholic acid, β-muricholic acid (β-MCA), and UDCA in double-inoculated mice, but the concentration of UDCA was lower than DCA (Supplemental Figure 4A). It has been reported that tauro-α (Tα) plus β-MCA increased by many fold in germ-free mice (37, 38). Consistent with these reports, we showed that germ-free mice inoculated with either *L*. *plantarum* or *C*. *scindens* had much higher serum Tα plus β-MCA levels compared with specific pathogen–free (SPF) mice; although double inoculations significantly reduced serum Tα plus β-MCA levels, they were still higher than that of SPF mice (Supplemental Figure 4B). It has been reported that muricholic acids are farnesoid X receptor (FXR) antagonists (39), making them less likely to be involved in the regulation of Rsp3 gene expression. We also found that tauro-cholic acid levels tended to decrease with double inoculations, but not statistically so (Supplemental Figure 4C). Taken together, these data indicate that an HFD induces microbial changes, including enrichment of Lachnospiraceae and Ruminococcaceae, resulting in increased secondary BA production and subsequent gene upregulation of the Rspo3–LGR system in the colon.

The article "Secondary bile acids mediate high-fat diet–induced upregulation of R-spondin 3 and intestinal epithelial proliferation" was retracted in 2024. Reasons: fabricated or falsified data; an official misconduct investigation.

### DCA increased Rspo3 gene expression via membrane receptor TGR5 in myofibroblasts.

To investigate the underlying mechanisms by which BAs regulate Rspo3 gene expression, we isolated and cultured the primary myofibroblasts from rat colon according to the method reported by Khalil et al. (40). We first characterized the phenotype of the cultured cells. Myofibroblasts are defined as cells that are α-SMA positive, vimentin positive, and desmin negative (41); therefore, we performed triple immunofluorescence staining. Cells isolated and cultured from rat colon stained positive for both α-SMA and vimentin but negative for desmin, indicating that they are myofibroblasts (Figure 5A). These cells also stained positive for Rspo3 (Figure 5B), which was further confirmed by RT-PCR (Figure 5C). The primary myofibroblasts also expressed the membrane receptor of BAs, TGR5, and the nuclear receptor FXR-α (Figure 5C). Treatments of the myofibroblasts with the secondary BA DCA increased Rspo3 gene expression in a dose-dependent manner (Figure 5D). However, the primary BA, CA, showed no effect on Rspo3 expression. LCA had a double-phased effect on Rspo3 expression: at very low doses (0.1 to 1 nM/L), it stimulated Rspo3 gene expression, at ≥10 nM/L doses, it either had no effect or had a tendency to suppress Rspo3 expression (Supplemental Figure 6A). CDCA also stimulated Rspo3 gene expression, but it was less potent compared with DCA (Supplemental Figure 6B). These findings are consistent with the fact that secondary BAs, such as DCA, are a much more potent activator of TGR5 compared with primary BAs, such as CDCA and CA (42), and LCA is more toxic to the liver (43).

The article "Secondary bile acids mediate high-fat diet–induced upregulation of R-spondin 3 and intestinal epithelial proliferation" was retracted in 2024. Reasons: fabricated or falsified data; an official misconduct investigation.

Because BAs can activate both the membrane receptor TGR5 and the nuclear receptor FXR-α, we next investigated which receptor mediates the upregulation of Rspo3 gene expression induced by BAs. We treated the myofibroblasts with either the TGR5-specific agonist oleanolic acid or the nuclear receptor FXR-α–specific agonist GW4064. Oleanolic acid stimulated Rspo3 gene expression, whereas GW4064 had no effect (Figure 5E). Moreover, knockdown of TGR5 abolished DCA-stimulated Rspo3 gene expression in the myofibroblasts (Figure 5E). Quantitative PCR showed that TGR5 was decreased by 60% after knockdown (Figure 5F). These data indicate that DCA-induced upregulation of Rspo3 is mediated by TGR5.

### Rspo3 mediates HFD-induced intestinal proliferation.

Both an HFD and Rspos promote proliferation of the intestinal epithelium (5, 23, 44). We next investigated whether Rspo3 may mediate HFD-induced intestinal proliferation. We performed in vivo studies and showed that an HFD promoted BrdU incorporation into the intestinal crypts in the colon (Figure 6A) and ileum of mice (Figure 6B), compared with mice fed regular chow. Increased incorporation of BrdU into crypts induced by an HFD were prevented by concurrent treatment with cholestyramine. Similarly, immunofluorescent staining of Ki67, a marker for proliferation, was increased by 80% in the crypts of mouse colon after HFD feeding; proliferation was prevented by cholestyramine treatment (Figure 7A). However, staining of the differentiation marker CK20 was unchanged by either an HFD or concurrent cholestyramine treatment (Figure 7B).

To show that the upregulation of Rspo3 is responsible for intestinal proliferation evoked by an HFD, we developed an Rspo3 conditional KO mouse model by crossing Cre-ER mice with flox-Rspo3 mice to obtain Cre-ER/floxRspo3 mice. These mice were treated with i.p. injection of tamoxifen for 5 consecutive days; 2 weeks later, proliferation studies were performed. Tamoxifen treatment of Cre-ER/floxRspo3 mice resulted in an 80% to 90% reduction of Rspo3 gene expression in the colon (Supplemental Figure 7). Deletion of Rspo3 abolished the increase of HFD-induced BrdU incorporation and elevation of Ki67 staining in the mouse colon (Figure 7, C and D). Moreover, deletion of Rspo3 abolished DCA-induced BrdU incorporation in both colon and ileum (Figure 8, A and B). These data indicate that upregulation of Rspo3 is responsible for the increased intestinal epithelial proliferation after high-fat feeding.

The article "Secondary bile acids mediate high-fat diet–induced upregulation of R-spondin 3 and intestinal epithelial proliferation" was retracted in 2024. Reasons: fabricated or falsified data; an official misconduct investigation.

## Discussion

Obesity and HFD are known inducers of LGR5^+^ intestinal stem cells and promotors of colorectal cancer. Although epidemiologic studies have increasingly suggested a causal relationship between obesity and increased risk for colorectal cancer, discovering the mechanisms facilitating this increased risk has been elusive. In this study, we showed that Rspo3 is the main subtype of Rspo in the small and large intestines and is produced primarily by myofibroblasts beneath the intestinal crypts, findings that are consistent with a previous report that Rspo3 is highly expressed in pericryptal myofibroblasts in the lamina propria (45). We further demonstrated that intestinal Rspo3, LGR4, LGR5, and β-catenin levels were increased in response to HFD; the increase was mediated by enrichment of bacteria with prominent BA metabolic capability and resultant increased levels of secondary BAs. Elevated levels of Rspo3 subsequently acted on LGR4 and LGR5, resulting in upregulation of β-catenin, suggesting the enhancement of the Wnt/β-catenin signaling pathway and intestinal epithelial proliferation.

An HFD has been shown to enhance intestinal stem cell proliferation (11). Rspo plays a critical role in regulating intestinal stem cell homeostasis by potentiating Wnt/β-catenin signaling via LGR-dependent and LGR-independent pathways (8, 46). For the LGR-dependent pathway, when Rspo is absent, 2 specific plasma membrane–associated E3 ubiquitin ligases, zinc and ring finger 3 and ring finger protein 43 (RNF43), induce the internalization and degradation of the Wnt receptor FZD. In the presence of Rspo, Rspo binds to ZNFR3/RNF43 and LGR simultaneously, and this binding complex inhibits the ubiquitin E3 ligase activities of ZNFR3/RNF43, resulting in accumulation of the FZD receptor and activation of Wnt /β-catenin pathway via the inhibition of glycogen synthase kinase 3β activity (46). Precise control of Wnt signaling activity is vital for intestinal cell homeostasis and is tightly regulated. Rspos are key regulators of the canonical Wnt signaling pathway by acting as ligands for LGRs to amplify Wnt signaling activity (24). Wnt pathway hyperactivation is a conserved hallmark of intestinal cancer and is seen in a vast majority of colorectal cancers (47). Although the majority of colorectal cancers are due to *Apc* gene mutations (48), approximately 10% of colorectal cancers have gain-of-function mutations in Rspo, leading to upregulation of Wnt signaling (25). Furthermore, increased expression of Rspo3 enhanced Wnt/β-catenin signaling pathways in both Lgr5^+^ and Lgr4^+^ cells and resulted in intestinal tumorigenesis (44).

The article "Secondary bile acids mediate high-fat diet–induced upregulation of R-spondin 3 and intestinal epithelial proliferation" was retracted in 2024. Reasons: fabricated or falsified data; an official misconduct investigation.

Our results show that an HFD for 2 weeks resulted in marked upregulation of Rspo3 in the small intestine and colon of rodents. This increase in Rspo3 levels is likely mediated by diet-induced changes in the gut microbiota. We found that an HFD resulted in marked enrichment of Firmicutes populations and a reduction of Bacteroidetes, which is consistent with previous reports (49, 50). HFDs rapidly shift the gut microbial structure toward bile-resistant taxa, with increased BA production, particularly secondary BAs (51). This is consistent with our data showing HFD-induced enrichment of certain microbial taxa, particularly Lachnospiraceae and Ruminococcaceae. These bacterial families are known to be enriched with BA enzymes important in conversion of primary to secondary BAs (30, 52). In genetically susceptible *Kras*-mutant mice, an HFD induces changes in the microbial composition and promotes intestinal tumorigenesis independent of obesity (53). Fecal transplants from HFD-fed mice with intestinal tumors were able to transmit disease even in the absence of an HFD, whereas treatment with antibiotics blocked tumor progression. It has been reported that serum levels of DCA are increased by an HFD and reduced by antibiotic treatment in mice (31, 54), findings that provide a functional link between the gut microbiota and luminal BAs in the regulation of Rspo3 expression. To demonstrate a causal relationship between alteration of gut microbiota and upregulation of Rspo3, we showed that in germ-free mice, 2 weeks of HFD feeding did not induce upregulation of Rspo3, LGR4, LGR5, or β-catenin genes. In contrast, 2 weeks after oral gavage of germ-free mice with fecal microbiota from mice fed HFD, there was an 80% upregulation of colon Rspo3. These findings suggest that gut dysbiosis and enhanced BA secretion likely mediate the HFD-induced upregulation of Rspo3 expression.

Among the various food components tested, we found that diets enriched in fat were the most potent inducers of Rspo3 expression in the colon. This was followed by red meat and protein, whereas a diet high in carbohydrate had no effect on Rspo3 expression. These findings reflect the efficacy of these foods, particularly fat, in stimulating BA secretion (55, 56). We showed that concurrent administration of cholestyramine with an HFD prevented upregulation of Rspo3 levels in the colon, which verified BAs are involved in the regulation of Rspo3 expression. We further demonstrated that oral administration of DCA, a major secondary BA, increased Rspo3 gene expression in the colon in germ-free mice. Moreover, we showed that an HFD could only induce upregulation of Rspo3 in mice inoculated with both BSH-containing *L*. *plantarum* and 7α-dehydroxylase–containing *C*. *scindens*, resulting in elevated serum DCA levels, indicating that the transformation of primary to secondary BAs by gut microbiota is essential for HFD-induced upregulation of Rspo3. *L*. *plantarum* and *C*. *scindens* double inoculations in germ-free mice also elevated serum levels of UDCA, which is also a potent TGR5 agonist (57), suggesting that UDCA may also play a role in the upregulation of Rspo3 in these mice with HFD feeding. However, serum concentration of UDCA was not increased by an HFD in SPF mice, suggesting that it did not play a major role in HFD-induced upregulation of Rspo3 under normal physiological conditions. Involvement of secondary BAs in the regulation of Rspo3 expression in the gut is further confirmed by our in vitro studies showing treatment of the myofibroblasts with DCA increased Rspo3 gene expression. Taken together, these series of observations suggest that enrichment of gut microbiota, particularly with Lachnospiraceae and Rumincoccaceae, by an HFD results in increased metabolism of primary BAs into secondary BAs, which act to upregulate Rspo3 in gut myofibroblasts.

The article "Secondary bile acids mediate high-fat diet–induced upregulation of R-spondin 3 and intestinal epithelial proliferation" was retracted in 2024. Reasons: fabricated or falsified data; an official misconduct investigation.

Secondary BAs have been linked with increased risk for colorectal cancer (58–60). Authors of a recent meta-analysis of 8 geographically diverse cohorts found a core metagenomic signature for colorectal cancer, which included taxa enriched with 7α-dehydroxylation metabolic capacity, suggesting an association between HFD, elevated secondary BAs, and colorectal cancer (61). Secondary BAs have been shown to induce colonic stem cells and colonic epithelial proliferation by inducing Wnt/β-catenin signaling pathways (62). Yoshimoto et al. (54) also reported HFD-induced gut microbial changes and increased secondary BAs in a mouse model of hepatocellular carcinoma. Although our results suggest that BAs act via TGR5 receptors to induce Rspo3, resulting in enhancement of the Wnt pathway, a prior study showed that BAs acting on FXR was responsible for Lgr5^+^ stem cell function (63). However, an Apc^min/+^ mouse model of colorectal cancer was used in that study, which may explain the discordant results seen with our respective studies, because Apc and Rspo mutations have been shown to be mutually exclusive (25). Although a recent publication also suggested that BAs stimulate intestinal stem cell proliferation via activation of TGR5 (64), it is plausible that increased secondary BAs induced by an HFD may promote intestinal stem cell proliferation and tumorigenesis by either TGR5/Rspo–dependent or FXR/Rspo–independent mechanisms.

The article "Secondary bile acids mediate high-fat diet–induced upregulation of R-spondin 3 and intestinal epithelial proliferation" was retracted in 2024. Reasons: fabricated or falsified data; an official misconduct investigation.

In conclusion, our studies indicate that Rspo3 is the major subtype of Rspo in the gut and is mainly produced by myofibroblasts beneath the crypts. Our results highlight the role of an HFD in inducing changes in the gut microbial structure and increased secondary BA metabolism, resulting in increased Rspo3 levels and enhancement of the Wnt signaling pathway, leading to increase in epithelial proliferation. It is conceivable that over the long term, this upregulation of Wnt signaling may lead to colonic neoplasm.

## Methods

### Animal and tissue preparation.

Experiments were performed on male Sprague-Dawley rats (150 to 180 g; Charles River Laboratories) and C57BL/6 mice (18 to 20 g; Jackson Laboratory). The animals were housed 3/cage in a pathogen-free or germ-free facility with a 12-hour light/12-hour dark cycle. All the germ-free mouse experiments were performed at the University of Michigan Germ-Free Mouse Facility. Mice were given food and water ad libitum and allowed to acclimate in the facility for 2 days before being randomly assigned to dietary treatments.

Rats and mice were fed different diets for 2 consecutive weeks: either a control diet of regular chow (13.5% kcal fat), an HFD (58% kcal fat; D12330, Research Diets), or an HFD mixed with 6% (wt/wt) cholestyramine. For the antibiotic treatment group, rats were given ampicillin (1 g/L), vancomycin (500 mg/L), neomycin sulfate (1 g/L), and metronidazole (1 g/L) in drinking water while feeding on an HFD (29). At the conclusion of the 2 weeks, the animals were euthanized with CO_2_, and small and large intestines were harvested.

### Reagents and bacteria.

CA, CDCA, DCA, LCA, and cholestyramine resin were purchased from Sigma-Aldrich; BrdU was purchased from Roche. *L*. *plantarum* (ATCC 10241, strain designation: BUCSAV 248) and *C*. *scindens* (ATCC 35704, strain designation: VPI 13733) were purchased.

### RT-PCR and qPCR.

Total RNA of mouse and rat intestines was isolated using Trizol reagent (Invitrogen) and cleaned up with RNeasy kit (QIAGEN). RNA (4 μg) was transcribed into cDNA using oligo dT primers and superscript II (Invitrogen). Primers used in RT-PCR and qPCR are listed in Supplemental Tables 1 and 2. All primer pairs span 1 or more introns for both mouse and rat. Primers and probe sequences for *L*. *plantarum* and primers sequence for *C*. *scindens* were obtained from previous reports (65, 66). The PCR conditions were as follows: 95°C for 3 minutes, 1 cycle; 95°C for 30 seconds; 57°C for 30 seconds; 72°C for 1 minutes, 38 cycles; and 72°C for 10 minutes, 1 cycle with the GoTaq DNA polymerase (Promega). The PCR product was visualized in 1% agarose, and the PCR bands were cut out and purified with the QIAEX II Gel Extraction Kit (QIAGEN). The purified product was sent for sequencing. qPCR was performed using the Bio-Rad CFX-Connect Real-Time System using Fam-labeled probes or SYBR green.

The article "Secondary bile acids mediate high-fat diet–induced upregulation of R-spondin 3 and intestinal epithelial proliferation" was retracted in 2024. Reasons: fabricated or falsified data; an official misconduct investigation.

### ISH.

ISH was conducted using a modification of a previously described technique (67, 68). Mouse and rat Rspo3 cDNA fragments were generated by PCR from the hypothalamic cDNA libraries. α-SMA and vimentin were generated from colon cDNA libraries and subcloned into pBluescript SK, which has T3 and T7 RNA polymerase promoters (Stratagene). The cDNAs were confirmed by DNA-Seq. The Dig- or [^35^S]-labeled antisense and sense RNA probes were generated using standard in vitro transcription methodology (69).

Tissue sections were washed twice with 2× SSC and then digested with 0.45 g/mL proteinase K (Invitrogen) in 100 mM Tris, pH 8.0, 50 mM EDTA for 15 minutes at 37°C. The sections were briefly washed with distilled water and then acetylated with 0.25% acetic anhydride in 0.1 M triethanolamine, pH 8.0, for 10 minutes. The sections were subsequently dehydrated through a graded series of ethanol.

Antisense or sense probes were diluted in hybridization buffer (50% formamide, 3× SSC, 1× Denhardt’s solution, 200 g/mL yeast tRNA, 50 mM phosphate buffer, pH 7.4, 10% dextran sulfate, and 10 mM DTT) to yield 30,000 cpm/μL for [^35^S]-labeled probes, or 3 to 4 μL probes per 100 μL of hybridization buffer for Dig-labeled probes. A total of 50 μL diluted probes were applied to each slide and the sections were coverslipped. Slides were then placed in sealed plastic boxes lined with filter paper moistened with 50% formamide. The boxes were wrapped with plastic wrap and incubated at 55°C overnight. For dual-label ISH, the sections were hybridized with Dig- and [^35^S]-labeled probes.

Following overnight incubation, cover slips were removed by dipping in 2× SSC and the slides were washed once for 2 minutes with 2× SSC. Slides were then incubated with 40 g/mL RNase A (Roche) in 10 mM Tris-HCl, pH 8.0, with 0.5 M NaCl at 37°C for 1 hour. The slides were washed with 2×, 1×, 0.5×, and 0.1× SSC at room temperature for 5 minutes each time, then incubated in 0.1× SSC at 67°C for 1 hour. The sections were washed briefly with distilled water. For single [^35^S]-label ISH, the slides were dehydrated in graded alcohols and air-dried. Dried slides were exposed to Kodak BioMax film.

The article "Secondary bile acids mediate high-fat diet–induced upregulation of R-spondin 3 and intestinal epithelial proliferation" was retracted in 2024. Reasons: fabricated or falsified data; an official misconduct investigation.

For dual-label ISH, after washing with distilled water, the slides were incubated in block buffer (0.25% carrageenan, 0.5% Triton X-100, 0.1 M sodium phosphate buffer, pH 7.25) for 1 hour and then were incubated with anti-dig Ab (Roche catalog 11093274910) conjugated with alkaline phosphatase diluted (1:6,000) in blocking buffer overnight at room temperature. The slides were washed twice in 0.1 M sodium phosphate buffer, pH 7.25, 2 minutes each, and twice in Tris-buffered saline buffer (100 mm Tris-HCl, pH 7.5, 150 mm NaCl), 10 minutes each followed by incubation in alkaline substrate buffer (ABS; 100 mm Tris, pH 9.5, 150 mm NaCl, 50 mm MgCl_2_). For color reaction, the slides were incubated in ABS buffer containing nitro blue tetrazolium chloride/5-bromo-4-chloro-3-indolyl-phosphate mix, 20 μL/mL; 5% polyvinyl alcohol, and 0.24 mg/mL levamisole for 2 to 4 hours. The slides were then dehydrated and dipped in ILFORD K.5D nuclear emulsion and exposed in dark for 10 to 14 days at 4°C. Sections were developed with D-19 developer. Colocalization was defined as cluster of silver grains are at least 4 times higher in the cell over background.

### Immunofluorescence and IHC.

Immunofluorescence staining was performed against Rspo3, α-SMA, vimentin, desmin, Ki67, CK20, LGR4, LGR5, β-catenin, and BrdU. All the primary and secondary Abs used are listed in Supplemental Table 3. Briefly, the slides or sections were washed 3 times in wash buffer (PBS) and immersed in a blocking solution (5% normal serum similar to the source of secondary Ab, 1% BSA, and 0.5% Triton X-100 in PBS) for 20 to 30 minutes to inhibit nonspecific binding. The sections were then incubated in a humid chamber overnight at 4°C with primary Abs. After incubation, the sections were washed 3 times in PBS buffer and incubated for 1 hour at room temperature with fluorophore-conjugated secondary Abs. For negative controls, the primary antiserum was omitted. For BrdU incorporation study, BrdU was dissolved in 7 mM NaOH/PBS and injected (i.p.) in mice at the dose of 100 mg/kg. After 4 hours, the mice were euthanized, the intestines were fixed, and 6 μm sections were cut and stained using rat anti-BrdU Ab. BrdU^+^ cells were visualized using either biotinylated goat anti-rat Ab and avidin biotin complex HRP kit (PK4000, Vector Laboratories; IHC), or cy3-goat anti-rat secondary Ab (immunofluorescence).

### Isolation and culture of primary myofibroblasts from rat colon.

Myofibroblasts of rat colon were isolated and cultured as previously reported (40). Briefly, the epithelial cells were denuded with 5 mM EDTA in HBSS and digested in RPMI-5 (Gibco), 10 U of dispase (MilliporeSigma), and 2,000 U of collagenase D (MilliporeSigma). The resulting cells were passed through a 70 μm mesh strainer (Falcon, Corning), cells were cultured in dishes for 3 hours, followed by 2 washes with HBSS to gently wash off nonadherent cells. because macrophages and epithelial cells senesce after the first passage, only myofibroblasts remain 1 week after seeding. Fresh RPMI-5 was added to grow the cells in cell culture.

The article "Secondary bile acids mediate high-fat diet–induced upregulation of R-spondin 3 and intestinal epithelial proliferation" was retracted in 2024. Reasons: fabricated or falsified data; an official misconduct investigation.

### Conditional deletion of Rspo3.

Tamoxifen-inducible Cre-ER mice [B6.Cg-Tg(CAG-cre/Esr1)5Amc/J], and Rspo3^tm1.1Jcob^/J mice with *loxP* sites flanking exons 2 through 4 of the Rspo3 gene were purchased from Jackson Laboratory. The Cre-ER mice were crossed with flox-Rspo3 mice, resulting in Cre-ER/floxRspo3 mice. Injection of tamoxifen (100 mg/kg, i.p.) (MilliporeSigma) for 5 consecutive days resulted in the deletion of exons 2 through 4 of *Rspo3* gene, which encode the furin-like and TSR-1 domains of Rspo3. Two weeks later, BrdU incorporation studies were performed as described above.

### Bacterial DNA isolation.

Bacterial genomic DNA was extracted by using a modified protocol of the QIAGEN DNeasy Blood & Tissue Kit. These modifications included (i) adding a bead-beating step using UltraClean fecal DNA bead tubes (Mo Bio Laboratories, Inc.) that were shaken using a Mini-Beadbeater-16 (BioSpec Products, Inc.) for 1.5 minutes, (ii) increasing the amount of buffer ATL used in the initial steps of the protocol (from 180 μL to 360 μL), (iii) increasing the volume of proteinase K used (from 20 μL to 40 μL), and (iv) decreasing the amount of buffer AE used to elute the DNA at the end of the protocol (from 200 μL to 85 μL).

### MiSeq Illumina sequencing.

Samples were submitted to the University of Michigan Medical School Host Microbiome Initiative and processed using the MiSeq Illumina sequencing platform. Primers specific to the V4 region were used to construct 16S rRNA gene libraries.

### OTU assignment and diversity measurements.

Sequences were curated using the community-supported software program *mothur* (version 1.39) (70) following the steps outlined in the MiSeq SOP (71). Sequences were assigned to OTUs using a cutoff of 0.03 and classified against the Ribosomal Database Project 16S rRNA gene training set (version 9) using a naive Bayesian approach with an 80% confidence threshold. Curated OTU sequence data were converted to relative abundance ± SEM. Within-community diversity (α-diversity) was calculated using the Shannon diversity index (H′) and OTU richness. Between-community diversity (β-diversity) was determined using the Yue and Clayton (θ_YC_) dissimilarity distance metric. Nonmetric multidimensional scaling was used to ordinate the β-diversity data. An analysis of molecular variation was used to test for significant differences in community structure using 10,000 permutations. To test for OTUs that were differentially abundant, biologically consistent, and having the greatest effect size, we used linear discriminant analysis effect size (multiclass = 1 vs. 1) (72).

The article "Secondary bile acids mediate high-fat diet–induced upregulation of R-spondin 3 and intestinal epithelial proliferation" was retracted in 2024. Reasons: fabricated or falsified data; an official misconduct investigation.

### BA measurement.

BAs in mouse serum were quantified at the University of Michigan Metabolomics Core. Briefly, after 2-step extraction, supernatants were combined, dried, and resuspended for liquid chromatography–mass spectrometry separation by reverse-phase liquid chromatography and measured using ESI-QQQMRM methods (73).

### Statistics.

All results are shown as mean ± SEM for the number of rats or mice indicated. For statistical analyses, unpaired 2-tailed Student’s *t* test and 1-way ANOVA with Bonferroni post hoc analysis were used. *P* < 0.05 was considered significant.

### Study approval.

All procedures were performed in accordance with NIH guidelines and were approved by the University of Michigan Committee on Use and Care of Animals.

## Author contributions

JYL designed and performed the experiments, analyzed the data, and wrote the manuscript. CO designed the experiments, analyzed the data, made critical revisions of the manuscript for important intellectual content, and obtained funding. MG performed the experiments, analyzed the data, and edited the manuscript. AAL reviewed the data and revised the manuscript. XW and SYZ performed the experiments and analyzed the data.

## Supplementary Material

Supplemental data

## Figures and Tables

**Figure 1:** Rspo proteins were detected in intestine and intestinal myofibroblasts by RT-PCR and ISH. RT-PCR of Rspo proteins 1 through 4 in the intestine of mouse (**A**), rat (**B**), and human colon and organoids (**C**). (**D**) Microphotograph of Rspo3 ISH in rat ileum. Clusters of silver grains representing Rspo3 mRNA are located beneath the crypts (left). Negative control was performed using Rspo3 sense probe (right). Double ISH shows that Rspo3 (silver grains) colocalized with α-SMA (purple), a marker for myofibroblasts, which was located beneath the crypts in (**E**) rat ileum and (**F**) colon. (**G**) Rspo3 colocalized with vimentin, a marker for fibroblasts, in rat colonic lamina propria. (**H**) Rspo3 colocalized with α-SMA underneath the crypts in mouse colon. Colocalization was defined as a cluster of silver grains overlapped with purple color. *n* = 3.

**Figure 2:** An HFD promotes upregulation of Rspo3, LGR4, LGR5, and β-catenin gene expression. (**A**) An HFD increased gene expression of Rspo3, LGR4, LGR5, and β-catenin in mouse colon, as determined by qPCR. Gene expression was normalized to the expression level of GAPDH. *n* = 5 or 6. (**B**) In mouse colon, Rspo3 gene expression was also upregulated by diets high in protein and red meat but not by a high-carbohydrate diet. *n* = 6. (**C**) In rat colon, the expression of Rspo3, LGR4, LGR5, and β-catenin were upregulated by an HFD but reversed by concurrent feeding with the BA binder, cholestyramine (6%), with HFD. *n* = 5 to 10. (**D**) In germ-free mice, an HFD did not increase gene expression of Rspo3, LGR4, LGR5, or β-catenin in the colon. *n* = 5. (**E**) Conventionalization of germ-free mice with regular mouse fecal microbiota increased Rspo3 mRNA in the colon. *n* = 5. (**F**) Broad-spectrum antibiotics (ampicillin, 1 g/L; vancomycin, 500 mg/L; neomycin sulfate, 1 g/L; and metronidazole, 1 g/L in drinking water) reversed the effects of an HFD on Rspo3 in rat colon. *n* = 5. For statistical analysis, a 2-tailed unpaired Student’s *t* test (**A**, **B**, and **D**) or 1-way ANOVA with Bonferroni post hoc analysis (**C**, **E**, and **F**) was used. *P < 0.05, **P < 0.01. In all plots, data are shown as the mean ± SEM. Abx, antibiotics; Carb, carbohydrate; RC, regular chow.

The article "Secondary bile acids mediate high-fat diet–induced upregulation of R-spondin 3 and intestinal epithelial proliferation" was retracted in 2024. Reasons: fabricated or falsified data; an official misconduct investigation.

**Figure 3:** The BA binder, cholestyramine (6% mixed in food), treatment prevented HFD-induced dysbiosis in rats. Differentially abundant OTUs (**A**, 1 to 20; **B**, 21 to 38) that were significantly enriched by HFD and reversed by cholestyramine treatment. Linear discriminant analysis effect size was used to determine which OTUs were differentially abundant (*P* < 0.05). *n* = 4 to 6.

**Figure 4:** Antibiotics treatment prevented HFD-induced dysbiosis. Differentially abundant OTUs (**A**, 1 to 20; **B**, 21 to 40) that were significantly enriched by HFD and reversed by Abx treatment. For the Abx treatment, rats were given ampicillin (1 g/L), vancomycin (500 mg/L), neomycin sulfate (1 g/L), and metronidazole (1 g/L) in drinking water while eating an HFD. Linear discriminant analysis effect size was used to determine which OTUs were differentially abundant (*P* < 0.05). *n* = 5. RC, regular chow.

**Figure 5:** Secondary BAs increased Rspo3 gene expression in myofibroblasts via TGR5. (**A**) Primary myofibroblasts from rat colon stain positive for α-SMA and vimentin, and negative for desmin. (**B**) Myofibroblasts stain positive for α-SMA, vimentin, and Rspo3. (**C**) RT-PCR of Rspo3, BA membrane receptor TGR5, and nuclear receptor FXR-α and pregnane X (PRX) in primary myofibroblasts. (**D**) Secondary BA DCA, but not primary BA CA, increased Rspo3 gene expression in myofibroblasts. *n* = 6. (**E**) TGR5-specific agonist oleanolic acid (1 μM/L) increased Rspo3 gene expression, but the nuclear receptor–specific agonist GW4064 (1 μM/L) had no effect (left). Knockdown of TGR5 abolished the effect of DCA on Rspo3 expression (right). *n* = 5. (**F**) qPCR showed that TGR5 was decreased by 60% after knockdown. *n* = 5. One-way ANOVA with Bonferroni post hoc analysis (**D** and **E**) or 2-tailed unpaired Student’s *t* test (**F**) was used. *P < 0.05, **P < 0.01.

The article "Secondary bile acids mediate high-fat diet–induced upregulation of R-spondin 3 and intestinal epithelial proliferation" was retracted in 2024. Reasons: fabricated or falsified data; an official misconduct investigation.

**Figure 6:** Cholestyramine treatment prevented HFD-induced BrdU incorporation into intestinal crypts. BrdU IHC of mouse colon (**A**) and ileum (**B**) showing BrdU incorporation into crypts in the group of regular chow, HFD, or HFD plus cholestyramine. Data are summarized in bar graphs. One-way ANOVA with Bonferroni post hoc analysis was used to compare groups. *P < 0.05. *n* = 5.

**Figure 7:** Rspo3 mediates HFD-induced intestinal proliferation. (**A**) Immunofluorescence of Ki67, a marker for proliferation, in mouse colon in the group fed regular chow (RC), HFD, or HFD plus cholestyramine. Data are summarized in bar graphs. *n* = 4. (**B**) Immunofluorescence of CK20, a marker of differentiation, in mouse colon in the same groups of mice. *n* = 4. (**C**) BrdU IHC in mouse colon in the groups of WT, RC; WT, HFD; and Rspo3 KO, HFD mice. Data are summarized in bar graphs. *n* = 3. (**D**) Immunofluorescence of Ki67 in the colon of the same groups of mice. *P < 0.05. *n* = 3. One-way ANOVA with Bonferroni post hoc analysis was used to compare groups.

**Figure 8:** Rspo3 mediates DCA-induced intestinal proliferation. BrdU immunofluorescence of mouse colon (**A**) and ileum (**B**) in the group of WT, WT plus DCA (0.15% in drinking water), or Rspo3 KO plus DCA. Data are summarized in bar graphs. One-way ANOVA with Bonferroni post hoc analysis was used to compare groups. **P < 0.01. *n* = 6.

## Version 1 09/13/2022

In-Press Preview

## Version 2 10/10/2022

Electronic publication
